# Antimicrobial activities of different solvent extracts from stem and seeds of *Peganum Harmala* L

**DOI:** 10.1371/journal.pone.0265206

**Published:** 2022-04-28

**Authors:** Muhammad Arif, Xiukang Wang, Mohammad Sayyar Khan Kazi, Shahid Ullah Khan, Sumbul Saeed, Amir Muhammad Khan, Rahmat Ali Khan, Masood Afzal, Ayesha Fazal Nawaz, Muhammad Amir Zia, Hosam O. Elansary, Shadi Shokralla, Abdullah Alhalabi, Alia Gul, Sajid Fiaz

**Affiliations:** 1 Faculty of crop production sciences, Institute of Biotechnology and Genetic Engineering (IBGE), The University of Agriculture, Peshawar, Khyber Pakhtunkhwa, Pakistan; 2 Department of Biotechnology, University of Mianwali, Mianwali, Punjab, Pakistan; 3 Key Laboratory of Protein Sciences, Department of Plant Biology and Ecology, College of Life Sciences, Nankai University, Tianjin, China; 4 College of Life Sciences, Yan’an University, Yan’an, Shaanxi, China; 5 Department of Biochemistry, Women Medical and Dental College, Abbottabad, KPK, Pakistan; 6 College of Plant Science and Technology, Huazhong Agricultural University, Wuhan, China; 7 Department of Botany, University of Mianwali, Mianwali, Pakistan; 8 Department of Biotechnology, University of Science and Technology, Bannu, KP, Pakistan; 9 Department of Chemistry, University of Mianwali, Mianwali, Punjab, Pakistan; 10 National Institute for Genomics and Advanced Biotechnology (NIGAB), National Agriculture Research Council, Islamabad, Pakistan; 11 Plant Production Department, College of Food and Agriculture Sciences, King Saud University, Riyadh, Saudi Arabia; 12 Centre for Biodiversity Genomics, University of Guelph, Guelph, ON, Canada; 13 School of Agriculture, Food and Wine, The University of Adelaide, Adelaide, Australia; 14 Department of Botany, Hazara University, Mansehra, Pakistan; 15 Department of Plant Breeding and Genetics, The University of Haripur, Haripur, Pakistan; Anhui Agricultural University, CHINA

## Abstract

Wild medicinal herbs have been used as folk and traditional medicines all across the world since well before recorded history. This present study was designed to test the antimicrobial activities of five different solvent extracted samples (*n-hexane*, *n-butanol*, *ethyl acetate*, *methanol*, and *water*) of *Peganum harmala* using stems and seeds. Two different strains of Gram-negative bacteria (*Escherichia coli* and *Klebsiella pneumonia)*, two Gram-positive bacteria *(Bacillus subtilus* and *Staphylococcus aureus)*, and one fungal strain (*Candida albicans*) were used. The antimicrobial activities were measured using a disc diffusion assay. Two concentrations of the extracts (1 and 2mgDisc^-1^) were used. *Ethyl acetate* fraction was found more affective among the tested solvents and showed maximum activity (zone of inhibition) against *S*. *aureus (*65.53 and 81.10%*)*, *E*. *coli (*46.22 and 61.29%*)* while *n-butanol* and *water* fractions gave maximum activity against *S*. *aureus* (78.86 and 70.00%) *and K*. *pneumonia* (57.00 and 61.39%) respectively. *Water* fraction showed maximum activity against *C*. *albicans* (60.00 and 81.88%). In the case of the stem, *Ethyl acetate* again showed more activity against *B*. *subtilus* (38.57 and 42.10%) and S. *aureus* (36.66 and 46.66%) while *n-butanol* showed maximum activity against *K*. *pneumonia* (24.55 and 32.44%) and *E*. *coli* (27.93 and 37.61%). *Methanol* was found more effective against *C*. *albicans* (25.71 and 43.80%). Seed extracted samples were found more effective compared to the stem. *Ethyl acetate*, *butanol*, and *aqueous* extracted samples showed good activity against the tested microbes, so these fractions are recommended for study their mechanism of actions and isolation of bioactive metabolites responsible for antimicrobial activities. The *P*. *harmala* should be evaluated for their bioactive compounds to be used in future studies. Our objective is to provide the framework for future study on the roles of *P*. *harmala* as traditional medicines.

## 1. Introduction

Our environment is teeming with harmful germs, and plants and animals are vulnerable to infection [1]. Attempts are being undertaken in a variety of ways to prevent and control these diseases. Natural herbal plants have historically been utilized to treat a range of diseases, either directly or indirectly through their bioactive metabolites [2]. The unrivaled chemical variety of natural products, whether as pure chemicals or as standardized plant extracts, provides unlimited possibilities for new medicine development [3]. Researchers are increasingly turning to folk medicine for new ideas on how to develop stronger antibiotics for microbial illnesses [4]. The urge to evaluate the antibacterial activity of medicinal plants arose in response to the increasing failure of chemotherapeutics and antibiotic resistance exhibited by pathogenic microorganisms. Since the beginning of time, man has used a variety of plants and their diverse components to avoid and treat various illnesses [5,6].

According to a World Health Organization (WHO) research, medicinal plants are utilized for basic health care by 80% of the world’s population [7]. Since ancient times, herbal plants have been used in various health remedies globally. Medicinal plants have a wide range of bioactive compounds that can be used to treat chronic and infectious diseases [8]. To assess the efficacy of medicinal plants, evidence from places where they are still used as medicine must be obtained. Alkaloids, flavonoids, tannins, and phenolic acids are the most important physiologically active compounds in medicinal plants, and they have physiological effects on the human body. These plants are well known as traditional medicines in rural areas of many poor countries [9]. Traditional therapists think that treatment derived from medicinal plants is more effective and less expensive than modern pharmaceuticals. In underdeveloped countries, low-income people, such as farmers and people from small villages, frequently use traditional medicine to treat common ailments [2,10,11].

*Peganum harmala* L belongs to family *Zygophylaceae* is a species of *Peganum*, also known as Alharmal, is one of the most valuable medicinal herbs [2,12]. Its many components are used in traditional medicine to treat a number of human illnesses, including lumbago, asthma, colic, jaundice, and as an emmenagogue stimulant [13]. It is a glabrous perennial herbaceous plant that thrives in semi-arid range terrain and sandy soils predominantly around the globe [4,6]. It can grow to a height of 0.8 meters. Alkaloids, flavonoids, and anthraquinones (antimalarial) are some of the well-known phytochemicals found in *P*. *harmala* [14,15]. It contains up to 4% total alkaloids [1]. *P*. *harmala* L has been demonstrated in several studies to have pharmacological and biological characteristics such as antibacterial, antifungal, and monoamine oxidases (MAO) [16].

*P*. *harmala* has anti-carcinogenic, vasodilator, anti-protozoal, and anti-inflammatory effects [1,17,18]. People in West Asia used to burn *P*. *harmala* seeds to produce smoke that protected them from voodoo [19]. Because of their analgesic and antibacterial properties, their fruits are used in traditional medicine. *P*. *harmala* has traditionally been used in traditional medicine to treat a wide range of conditions, including hepatitis B, asthma, lumbago, and colic [15]. The hallucinogenic -carboline alkaloids harmine, harmaline, harmalol, harmalacinine, isoharmin, and 8-glucosyloxyharmine are discovered in seeds [20]. Smoke is used as a disinfectant, an air cleaner, and a cold remedy. Research revealed the chemical composition and antibacterial activity of this smoke, however, the technique and temperature used to produce and analyze the smoke were still not clear [21].

However, little work has been done on phytochemical extracts as far as antimicrobial activities are concerned. Here we have focused on antimicrobial activities of different solvent extracts such as *n-hexane*, *n-butanol*, *ethyl acetate*, *methanol*, and *wate*r of *P*. *harmala* using stem and seeds by disc diffusion method. *Ethyl acetate* fraction was found more effective among the tested solvents and showed maximum activity against *Staphylococcus aureus* and *Escherichia coli* while *n-butanol* and *water* fractions gave maximum activity against *S*. *aureus and Klebsiella pneumonia* respectively. The *water* fraction has the greatest antifungal activity against *Candida albicans*. In the case of stem, *ethyl acetate* was more active against *Bacillus subtilis* and *S*. *aureus* while *n-butanol* was against *K*. *pneumonia* and *E*. *coli*. *Methanol* is more effective than *ethanol* against *C*. *albicans*. Seed extracts outperformed stem extracts in terms of efficacy. The extracted samples of *ethyl acetate*, *butanol*, and *water* have shown good antimicrobial activity against the tested bacteria, hence these solvents are recommended for future studies.

## 2. Materials and methods

### 2.1 Plant materials collection

The present study was conducted at the Institute of Biotechnology and Genetic Engineering (IBGE), University of Agriculture, Peshawar Pakistan. *P*. *harmala* seeds were bought from a local market in Bannu, Khyber Pakhtunkhwa, Pakistan. 200 grams seeds were collected and then were grown in pots at the greenhouse of IBGE. 4 plants per pot are grown and a total of 22 pots were prepared. Stems were collected to obtain extracts from growing plants. All the plants were healthy and used for further experimental work. Plant materials were washed and dried at room temperature.

### 2.2 Crude extract preparation

The dried plant components, both seed and stem were ground into a fine powder using a grinder. The powdered components were soaked in *methanol* for one week. During this period, the plant components were combined daily to ensure that the bioactive compounds were fully dissolved. The plant materials were filtered and dried under reduced pressure in a rotary evaporator (Lab Tech EV311H). The entire process was repeated three times, each time combining all fractions. After that, the extract was transferred to a separating funnel and blended with 250-300ml of distilled water. An exact amount of *n-hexane* was added, shaken, and allowed to stand for 5–10 minutes. The organic layer was collected, and the process was performed three times more, each time with the addition of a fresh organic solvent. A variety of fractions were separated by adding *n-butanol* and *ethyl acetate* to water one at a time. All of the organic layers were then dried at reduced pressure using a rotary evaporator (Lab Tech EV311H) [22].

### 2.3 Fractionation

Eight to ten grams of crude *methanolic* extract from both seed and stem samples were kept for biological/pharmacological activities. The remaining was dissolved in 300 ml distilled *water* and was shifted to a separatory funnel and then added 300 ml of *n-hexane*. Shaking of the separatory funnel was done to separate the two layers of *water* and *n-hexane*. The *n-hexane* fraction formed the upper layer as it is lighter than *water*. The upper *n-hexane* layer was collected and the second layer of *water* was fractioned two times more with *n-hexane*. All the fractions of *n-hexane* were collective, filtered through Whatman filter paper, and dried through the rotary evaporator to obtain *n-hexane* fraction. The same fractionation procedure was conceded for *ethyl acetate* and *n-butanol* to obtain its extracts. The *aqueous* layer at the end was desiccated using a rotary evaporator. In this way, crude methanol; *n-hexane*, *n-butanol*, *ethyl acetate*, and *aqueou*s fractions were obtained. A similar procedure was used for the stem parts also to get their extracts [22].

### 2.4 Media preparation for culturing

Nutrient agar media and nutrient broth were used during the study. Agar media was used for microbial culturing and growth while the nutrient broth was used for standardization and incubation (Tables 1 and 2). The required ingredients of the nutrient agar and nutrient broth were dissolved in distilled water and poured into conical flasks. All the media flasks and test tubes were sealed with cotton buds and then sterilized in an autoclave (Labtron) at 1.5 pounds pressure and 121°C temperature for 15 min. After sterilization, the media was poured into Petri plates under aseptic conditions in the laminar flow chamber. The plates were then stored in an incubator (BIOBASE Biodustry Shandong, china) at 37°C for 4 hours for later use. The nutrient broth in flasks (approximately 20 ml flask^-1^) was used for shaking incubation of microorganisms and nutrient broth in test tubes for standardization of microbial cultures [4,22].

**Table 1:** Composition of nutrient agar used for culturing of the tested microbes.

Nutrient Agar Modified QUELAB QB-39-3504	
Composition	g l^-1^
Beef extract	1
Yeast extract	2
Gelatin extract	5
Sodium chloride	5
Agar	15
Total	28

**Table 2:** Composition of nutrient broth used for shaking incubation and standardization.

Nutrient Agar Modified QUELAB QB-39-3504	
Composition	g l^-1^
Gelatin peptone	5
Beef extract	1
Yeast extract	2
Sodium chloride	5
Total	13

### 2.5 Microorganisms

Antimicrobial activity of different solvent extracted samples from seeds and stem of *P*. *harmala* was tested against four bacterial and one fungal strain (Table 3). All microbial stock cultures were freshened by streaking using a sterile inoculation loop on nutrient agar medium plates in a laminar flow hood (BIOBASE), incubated at 37°C for 24 hrs. After 24 hours, the streaked cultures were again sub-cultured on medium plates and incubated at 37°C for 24 hrs. The second streaked cultures were inoculated into nutrient broth in flasks and subjected to shaking incubation for 18 hours at 37°C (200 rpm). The selected bacterial and fungal strains for this study were *B*. *subtilis*, *K*. *pneumonia*, *S*. *aureus*, *E*. *coli*, and *C*. *albicans* (Table 3).

**Table 3:** Different microbial strains used during the experiment.

Microbial Species	Gram strain type	Details of the Microbial strains used
*Klebsiella pneumonia*	Negative	Clinical isolate obtained from Department of Microbiology, Quaid-I-Azam University Islamabad, Pakistan
*Staphylococcus aureus*	Positive	ATCC # 6538
*Bacillus subtilis*	Positive	Clinical isolate obtained from Department of Microbiology, Quaid-I-Azam University Islamabad, Pakistan
*Escherichia coli*	Negative	ATCC # 25922
*Candida albicans*	Fungal	ATCC#10231. Plant Pathology Department, The University of Agriculture, Peshawar KPK, Pakistan

### 2.6 Antibacterial and antifungal assay

The antibacterial activity of different solvent extracted samples of *P*. *harmala* was carried by disc diffusion assay as described in Bauer et al. 1966 and antifungal activity by Ramdas et al. 1998 against different bacterial and fungal strains [23,24].

### 2.7 Disc diffusion susceptibility method

Nutrient agar media plates were seeded with 18–24 hours cultures of microbial inoculums (a standardized inoculum 1–2 × 107 CFU ml-1 0.5 McFarland Standard). Whatman No. 1 filter paper discs (6 mm in diameter) were placed with the help of sterile forceps on the media and then plant extracts in concentrations of 1 and 2 mg disc-1 in 6 and 12μL volume were applied on the discs. Antibiotics (6 μL disc-1) as positive control and DMSO (6 μL disc-1) as negative controls were also applied on the discs. Inoculated plates were then incubated at 37°C for 18–24 hrs. The next day, zones of inhibition were recorded as an area in millimeters (mm) around the discs in each plate [4].

### 2.8 Positive controls

Erythromycin and ciprofloxacin were used as positive control for Gram-positive and Gram-negative bacteria. Clotrimazole was used as a positive control for fungal strain.

## 3. Results

### 3.1 *B*. *subtilis* response towards different extracts

The study was undertaken to evaluate the antimicrobial activities of different solvent extracted samples from stem and seed of *P*. *harmala* against four bacterial species including both gram-positive and gram-negative and one fungal species. *N-hexane*, *ethyl acetate*, *n-butanol*, *methanol*, and *aqueous* extracts from stem and seeds of *P*. *harmala* were tested against *B*. *subtilis* using disc diffusion assay (Fig 1). *B*. *subtilus* showed high susceptibility in the case of *n-butanol* and *ethyl acetate* extracted samples from stem extracted samples at lower and higher concentrations i.e. 1 and 2 mg discs^-1^. *N-butanol* extracted samples revealed the highest inhibitory activity (42.97% ZI) at a concentration of 2 mg disc^-1^. *Ethyl-acetate* extracted samples showed 42.10 percent inhibitory activity at 2 mg disc^-1^. *Methanol* showed 26.31 percent inhibitory activity at higher concentration i-e 2 mg disc^-1^, While 21.92% activity was shown at lower concentration i-e 1mg disc^-1^. *Aqueous* and *n-hexane* extracted samples showed the lowest activities (17.21% and 24.55% ZI respectively) at higher concentrations (2 mg disc-1) while lower concentrations (0 and 18.42% ZI) were observed (Fig 1). Compared with stem-derived extracts *n-butanol* and *ethyl acetate* again showed the highest activity in the case of seed extracted samples against *B*. *subtilus* at lower and higher concentrations i.e. 1 and 2 mg discs^-1^. *N-butanol* extracted samples revealed the highest inhibitory activity (57.00% ZI) at a concentration of 2 mg disc^-1^. *Ethyl-acetate* extracted samples showed 52.63 percent inhibitory activity at 2 mg disc^-1^. *Methanol* showed 57.89 percent inhibitory activity at higher concentration i-e 2 mg disc^-1^ and no activity was shown at lower concentration i-e 1mg disc^-1^. *N-hexane* and *aqueous* extracted samples showed the lowest activity (28.05% ZI each) at lower concentrations (1 mg disc^-1^) and (34.21% and 40.34% ZI) at higher concentrations compared with other samples (Fig 1).

**Fig 1:** Antimicrobial activity of n-hexane, ethyl acetate, n-butanol, methanol and water extracted samples from stem and seed of *Peganum harmala* against *Bacillus subtilis* by disc diffusion assay.

### 3.2 *K*. *pneumoniae* response towards different extracts

The same stem and seeds-derived extracts of *P*. *harmala* including *n-hexane*, *ethyl acetate*, *n-butanol*, *methanol*, and *aqueous* extracts were further tested against *K*. *pneumoniae*, using disc diffusion assay (Fig 2). It is clear from the data that *K*. *pneumoniae* was highly susceptible to *n-butanol* extracted sample both at 1 and 2 mg disc^-1^concentration. The *n-butanol* fraction showed the highest inhibitory zone (24.55% ZI at 1 mg disc^-1^ and 32.44% ZI at 2 mg disc^-1^). Similar activity was observed in the case of *n-hexane* and *aqueous* extracted samples (19.28%, 24.55%, and 15.78%, 27.18%). *Methanol* and *ethyl acetate* extracted samples though reduced the microbial growth i-e 13.15% and 21.92% and that of *ethyl acetate* is 14.02% and 18.42% respectively (Fig 2). Compared with stem extracted samples, seeds extracted samples showed good results. *K*. *pneumoniae* was highly susceptible to aqueous extracted samples both at 1 and 2 mg disc^-1^. The *aqueous* fraction showed the highest inhibitory zone (51.73% ZI at 1 mg disc^-1^ and 61.39% ZI at 2 mg disc^-1^). The *n-butanol* and *methano*l extracted samples revealed the same activity against *K*. *pneumoniae* (52.63% and 57.00% and 53.50% and 54.36% ZI for both *n-butanol* and *methano*l extracted sample) at 1 and 2 mg disc^-1^ respectively). *N-hexane* and *ethyl acetate* extracted samples though reduced the microbial growth i-e 35.94% and 38.07% and that of *ethyl acetate* is 40.34% and 52.63% respectively (Fig 2).

**Fig 2:** Antimicrobial activity of n-hexane, ethyl acetate, n-butanol, methanol and water extracted samples from stem and seed of *Peganum harmala* against *Klebsiella pneumoniae* by disc diffusion assay.

### 3.3 *S*. *aureus* response towards different extracts

The data regarding the antibacterial activity of *n-hexane*, *ethyl-acetate*, *n-butanol*, *methanol*, and *aqueous* extracted samples from the stem of *P*. *harmala* against *S*. *aureus* revealed that *S*. *aureus* is highly susceptible to all extracts of *P*. *harmala*. By increasing the concentration of different extracts, the degree of inhibition also increased. All the extracted samples were effective against *S*. *aureus* and inhibited the growth at both higher and lower concentrations (1 and 2 mg disc^-1^). *Ethyl acetate* extracted samples showed the highest inhibitory zones i.e. 46.66% at 2 mg disc^-1^ concentration. The lowest inhibitory zones were observed when *n-butanol* extracted samples were applied (22.20% at 2 mg disc^-1^) compared to a positive control (Fig 3). Comparing the antibacterial activity of *n-hexane*, *ethyl-acetate*, *n-butanol*, *methanol* and *aqueous* extracted samples from the seeds of *P*. *harmala* against *S*. *aureus* with stem extracted samples revealed that *S*. *aureus* is highly susceptible to all extracts of *P*. *harmala*. With increasing concentration of different extracts, an increased in the degree of inhibition was observed. *Ethyl acetate* extracted samples showed the highest inhibitory zones i.e. 81.10% at 2 mg disc^-1^ concentration. The lowest inhibitory zones were measured by *n-hexane* extracted samples (48.86% ZI at a concentration of 2 mg disc^-1^) when compared with positive controls (Fig 3).

**Fig 3:** Antimicrobial activity of n-hexane, ethyl acetate, n-butanol, methanol and water extracted samples from stem and seed of *Peganum harmala* against *Staphylococcus aureus* by disc diffusion assay.

### 3.4 *E*. *coli* response towards different extracts

The data regarding the antibacterial activity of *n-hexane*, *ethyl-acetate*, *n-butanol*, *methanol*, and *aqueous* extracted samples from the stem of *P*. *harmala* against *E*. *coli* by disc diffusion assay was also recorded (Fig 4). The data showed that all the solvent extracted samples gave significant activity. The *n-butanol* and *methanol* fraction reduced the growth of *E*.*coli* at both concentrations i-e 1mg and 2 mg disc^-1^ (27.93%, 37.61% and 23.64%, 35.48% respectively). Both *n-hexane* and *aqueous* extracted samples significantly reduced (33.32%) the growth of *E*. *coli* at higher concentrations. Compared with stem extracted samples, seeds extracted samples showed good activity except for *n-hexane* which did not restrict the growth of *E*.*coli*. The *ethyl acetate* and *aqueous* fraction reduced the growth of *E*.*coli* at both concentrations i-e 1 mg and 2 mg disc^-1^ (46.22%, 32.25% and 61.29%, 41.93% respectively). The *n-butanol* extracted samples significantly reduced the growth of *E*. *coli* i-e 56.96% ZI at a concentration of 2 mg disc^-1^ and no activity were shown on lower concentration i-e 1 mg disc^-1^, followed by crude methanolic extracted samples (53.74% ZI) at the highest concentration of 2 mg disc^-1^ and no activity were shown on lower concentration (Fig 4).

**Fig 4:** Antimicrobial activity of n-hexane, ethyl acetate, n-butanol, methanol and water extracted samples from stem and seed of *Peganum harmala* against *Escherichia coli* by disc diffusion assay.

### 3.5 *C*. *albicans* response towards different extracts

The data regarding the antifungal activity of *n-hexane*, *ethyl acetate*, *n-butanol*, *methanol*, and *water* extracted samples from the stem of *P*. *harmala* against *C*. *albicans* by disc diffusion assay showed that all five samples can reduce the growth of *C*. *albicans* at 1 and 2 mg/disc concentrations (Fig 5). Among these solvent extracted samples, *methanol* fraction showed the highest inhibitory activity (43.80%) at higher concentrations. Both n-*butanol* and *n-hexane* extracted samples reduced the growth of *C*. *albicans* (34.28% at the concentration of 2 mg per disc), while *ethyl acetate* and *aqueous* extracted samples showed the lowest inhibitory zones i.e 25.71% and 20.94% at higher concentration compared to positive control. Compared with stem extracted samples, in seeds extracted samples, the *aqueous* fraction showed the highest inhibitory zone i.e. 81.88% at 2 mg disc^-1^ concentration. *Ethyl acetate* and *methanol* extracted samples reduced the growth of *C*. *albicans* (78.08% and 74.28% at concentration of 2 mg per disc), while *n-butanol* and *n-hexane* extracted samples showed the lowest inhibitory zones i.e 59.02% and 40.00% at 2mg per disc as compared to a positive control (S1 Fig).

**Fig 5:** Antimicrobial activity of n-hexane, ethyl acetate, n-butanol, methanol and water extracted samples from stem and seed of *Peganum harmala* against *Candida albicans* by disc diffusion assay.

## 4. Discussion

Traditional medicines from various countries, which are the main source of complementary and alternative medicine, have recently shown promise in the treatment of a wide range of human diseases. The therapeutic approach of traditional medicine is heavily reliant on medicinal plants. *P*. *harmala* is a well-known medicinal plant with numerous pharmacological effects, including cardiovascular, neurologic, antimicrobial, anticancer, gastrointestinal, and antidiabetic properties. Several studies in modern phototherapy have confirmed some of the pharmacologic properties of this plant that have been documented in traditional Iranian medicine [16]. According to El-Saad El Rifaei, the compounds extracted from *P*. *harmala* plant have a variety of medical properties, including the anti-inflammatory effects of pitolin [25]. He confirmed antibacterial/antifungal, antifever, and antiparasitic effects in *P*. *harmala*. The majority of studies on *P*. *harmala* medical effects have concentrated on parasite infections. Levchenko was among the first to report on the medicinal properties of *P*. *harmala* alkaloids in bovines [20]. In this study, the antibacterial and antifungal activities of different solvent extracts were measured for bacterial and fungal strains by the disc diffusion method. The *ethyl acetate* fraction was found to be the most effective of the tested solvents, with maximum activity (zone of inhibition) against *S*. *aureus* (65.53 and 81.10%), *E*. *coli* (46.22 and 61.29%), and *K*. *pneumonia* (57.00 and 61.39%). Similar results were observed by Amel et al. (2012) [26]. They also used different solvent extracts against a wide-range of microorganisms. The same bacterial strains were reported by another group, and the antimicrobial activity was tested on 11 different bacteria using the agar diffusion method [27].

The water fraction had the highest activity against *C*. *albicans* (60.00 and 81.88%). In the case of the stem, *Ethyl acetate* was more effective against *B*. *subtilus* (38.57 and 42.10%) and S. *aureus* (36.66 and 46.66%) while n-butanol showed maximum activity against *K*. *pneumonia* (24.55 and 32.44%) and *E*. *coli* (27.93 and 37.61%). *Methanol* was found more effective against *C*. *albicans* (25.71 and 43.80%). Similar results were obtained by Hayet et al (2010) who also analyzed the antibacterial, antiviral and antioxidant activity of *P*. *harmala* against gram-positive and gram-negative bacteria [28]. These results are in contradiction with Dastagir and Hussain who have reported that the *n-hexane* extracts of *Zygophyllaceae* and *Euphorbiaceae* families showed the highest toxicity as compared to *methanolic* extracts [3]. Al-Izzy et al. (2010) also reported that the aqueous fraction from *P*. *harmala* was effective in the inhibition of the growth of these microorganisms [29].

## 5. Conclusion

*P*. *harmala*, a versatile traditional medicinal plant with a diverse range of bioactive compounds, is an abundant source of bioactive compounds. Because little research has been conducted on the biological activity and potential medicinal applications of phytochemical compounds. More research could result in the development of new high-potency medications. This study demonstrates *P*. *harmala* potential for usage in innovative therapeutic drugs and establishes the framework for future medicinal plant research and antibacterial activity of *P*. *harmala* extracts against drug-resistant/clinically significant microbes.

## Supporting information

S1 Fig Plate 1 and 2: Inhibition zone made by seed and stem extract of *Bacillus Subtilus* in *N-Butanol* solution where 1 indicate 6μl of diffused disc and 2 indicates 12μl, respectively. **Plate 3 and 4:** Inhibition zone made by seed and stem extract of *C*.*albicans* in water solution where 1 indicate 6μl of diffused disc and 2 indicates 12μl, respectively. **Plate 5 and 6:** Inhibition zone made by seed and stem extract of *K*. *pneumonia* in water solution where 1 indicate 6μl of diffused disc and 2 indicates 12μl respectively. **Plate 7 and 8:** Inhibition zone made by seed and stem extract of *E*.*Coli* in *Ethylacetate* solution where 1 indicate 6μl of diffused disc and 2 indicates 12μl respectively. **Plate 9 and 10:** Inhibition zone made by seed and stem extract of *S*. *aureus* in *Methanol* solution where 1 indicate 6μl of diffused disc and 2 indicates 12μl respectively.
(DOCX)

## Abbreviations

WHO: world health organization
P: harmala: Peganum harmala
S: aureus: Staphylococcus aureus
E: coli: Escherichia coli
K: pneumonia: Klebsiella pneumonia
B: subtilis: Bacillus subtilis
C: albicans: Candida albicans
ZI: zone of inhibition
